The article "NUCB2/Nesfatin-1 Regulation of Chronic Visceral Hyperalgesia" was retracted in 2023. Reasons: signs of a paper mill; compromised peer review; unreliable results or conclusions.

# NUCB2/Nesfatin-1 Regulation of Chronic Visceral Hyperalgesia

**DOI:** 10.1155/2022/4079533

**Published:** 2022-07-08

**Authors:** Qiaoyan Gu, Yuan Lei, Jianming Wu, Ting He, Juanjuan Li, Shanshan Song

**Affiliations:** Department of Gastroenterology, The Affiliated Hospital of Yan'an University, Yan'an Shaanxi Province, China

## Abstract

**Objective:**

We previously described that different concentration Nucleobindin-2 (NUCB2)/Nesfatin-1 gradients differently regulated visceral hypersensitivity in irritable bowel syndrome. Therefore, this study is aimed at evaluating the effect of NUCB2/Nesfatin-1 on model rats with chronic visceral hyperalgesia.

**Methods:**

Neonatal and mature Sprague-Dawley rats were randomly divided into the healthy control and chronic visceral hyperalgesia model groups. The model was built by combining maternal separation with the acetic acid enema. The models were identified by the distension volume threshold to reach abdominal withdraw reflex (AWR) score = 3, histological staining, and myeloperoxidase (MPO) detection. The visceral sensitivity to chronic visceral hyperalgesia was then evaluated.

**Result:**

Rats in the model group responded more strongly to pulling stimulation than healthy controls; the distension volume threshold causing AWR3 response in model rats was lower than the control group before NUCB2/Nesfatin-1 intervention. After intervention, the distension volume threshold was significantly lower in the NUCB2/Nesfatin-1 central intervention group than in the NUCB2/Nesfatin-1 peripheral intervention group, and the peak value of external oblique muscle electrical activity was significantly higher. Additionally, compared with the male intervention group, in the female intervention group, the volume threshold was significantly lower and the peak value was higher.

**Conclusion:**

NUCB2/Nesfatin-1 could regulate visceral sensitivity in chronic visceral hyperalgesia model rats; its regulatory effect correlated with the type of NUCB2/Nesfatin-1 intervention approaches (central or peripheral) and sex (male or female).

## 1. Introduction

Chronic visceral hyperalgesia is a pathological state of visceral paresthesia, one important biological and pathogenetic characteristic of irritable bowel syndrome (IBS). The sensitivity of chronic visceral hyperalgesia is closely connected to the fluctuation in clinical symptoms of patients with IBS [1–3]. An abnormal sensitization of peripheral and central sensory routes leads to the occurrence and development of chronic visceral hyperalgesia [4, 5]. An effective intervention and regulation of chronic visceral hyperalgesia is required for the prevention and treatment of IBS.

The article "NUCB2/Nesfatin-1 Regulation of Chronic Visceral Hyperalgesia" was retracted in 2023. Reasons: signs of a paper mill; compromised peer review; unreliable results or conclusions.

Nucleobindin-2 (NUCB2)/Nesfatin-1 is a multifunctional biomolecule, which plays an important role in the diagnosis and treatment of numerous diseases [6–9]. The in-depth study of NUCB2/Nesfatin-1 has shown its close relationship to IBS [10–12]. Our previous study showed that various NUCB2/Nesfatin-1 concentration gradients differently regulated visceral hypersensitivity in IBS [13]. Based on these studies, here, we built chronic visceral hyperalgesia models and administered NUCB2/Nesfatin-1 through different approaches; then, we compared the regulating effects of NUCB2/Nesfatin-1 on chronic visceral hyperalgesia sensitivity, laying the foundation for in-depth exploration of the relationship between NUCB2/Nesfatin-1 and IBS.

## 2. Materials and Methods

### 2.1. Animal and Materials

Neonatal (within 2 days, weight 1.8 g–6 g) and mature male and female Sprague-Dawley (SD) rats were purchased from the Research Department of Shanghai Family Planning Science. And the following materials were obtained: NUCB2/Nesfatin-1 (MedChemExpress, New Jersey, USA), myeloperoxidase (MPO) detection kit (Nanjing Jiancheng Bioengineering Institute, Nanjin, China), stereotaxie apparatus (Ruiwode, Shenzhen, China), and electrophysiological detector (Taimeng, Chengdu, China). Animal experiments were approved by the Animal Ethics Association of the Affiliated Hospital of Yan'an University (Ethics No. 2017-14).

### 2.2. Establishment of a Chronic Visceral Hyperalgesia Model

The model was developed in neonatal model rats from the 2nd to the 21st day after birth by combining maternal separation with an acetic acid enema. The rats were separated from their mothers for 3 h from 09:00 am to 12:00 am every day; during that time, breastfeeding was not possible. Then, from the 8th to the 20th day after birth, the rats received 0.3 mL 0.5% acetic acid at 02:00 pm through the anus once a day. The model intervention scheme ended on the 21st day. After completing the model intervention scheme, all rats in both the model group and healthy control group were weaned and maternal rats separated. The rats were then maintained in a standard environment with room temperature of 22°C–25°C, a relative humidity of 50%–60%, free drinking water, standard diet, and a 12 h day/night cycle for two weeks. After the growth adaptation period and the intestinal aseptic inflammation subsidation period, the model was validated [14–17].

### 2.3. Validation of the Chronic Visceral Hyperalgesia Model

We adopted the rat's abdominal withdrawal reflex (AWR) score as standard [17]; the distension volume threshold to reach AWR score = 3 (AWR3 response) was chosen to evaluate visceral sensitivity. The rats were sacrificed at the end of the experiment and two pieces of colonic tissue of 0.3–0.5 cm were isolated from the healthy group and the model group, respectively. Then, one piece of tissue was observed with the naked eye, fixed with formaldehyde solution, and hematoxylin-eosin (HE) staining was performed for pathological examination. The other piece of tissue was used to detect MPO activity by enzyme-linked immunosorbent assay. We combined histopathology analysis with MPO measurement to evaluate colon tissue inflammation.

The article "NUCB2/Nesfatin-1 Regulation of Chronic Visceral Hyperalgesia" was retracted in 2023. Reasons: signs of a paper mill; compromised peer review; unreliable results or conclusions.

### 2.4. Animal Groups and Intervention Scheme

Male (M group) and female (F group) rats in the healthy control group were fed in a standard environment after weaning. The male rats in the model group (*n* = 40) were randomly divided into five groups (*n* = 8 per group): the model control group (MC group), NUCB2/Nesfatin-1 central intervention group (MC+NCI group), central intervention control group (MC+SCI group), NUCB2/Nesfatin-1 peripheral intervention group (MC+NPI group), and peripheral intervention control group (MC+SPI group). Then, the MC+SCI and MC+NCI groups were injected with 0.5 *μ*L 0.9% normal saline (NS) and 0.5 *μ*L 50 *μ*mol/L NUCB2/Nesfatin-1 into the lateral ventricles, respectively; the MC+NPI and MC+SPI groups were injected with 0.5 *μ*L 0.9% NS and 0.5 *μ*L 50 *μ*mol/L NUCB2/Nesfatin-1 into the tail vein, respectively. After 2 h of adaptation, we evaluated the sensitivity of chronic visceral hyperalgesia in experimental rats.

The female rats in the model group (*n* = 40) were randomly divided into five groups (*n* = 8 per group): the MC group (FC group), NUCB2/Nesfatin-1 central intervention group (FC+NCI group), central intervention control group (FC+SCI group), NUCB2/Nesfatin-1 peripheral intervention group (FC+NPI group), and peripheral intervention control group (FC+SPI group). The intervention scheme was the same as the male chronic visceral hyperalgesia model group.

### 2.5. Measurement of Visceral Sensitivity

An 8Fr catheter with balloon was first inserted into the rats' anus. After the rats adapted and become quiet, 0.9% NS was injected into the balloon to dilate the rectum. The dilated balloon lasted for 10 s each time, every rat had to dilate the rectum 3 times at 4 min intervals. Then, we recorded the distension volume threshold causing AWR3 response and the peak value of external oblique muscle electrical activity and calculated the average value as an index to evaluate the sensitivity of chronic visceral hyperalgesia.

### 2.6. Statistical Analysis

All analyses were performed using the statistical package Empower (R) (http://www.empowerstats.com/; X&Y Solutions, Inc., Boston, MA). Data are presented as the mean ± standard deviation for continuous variables; the comparison of the different groups was performed by a one-way analysis of variance. *P* < 0.05 was considered statistically significant.

The article "NUCB2/Nesfatin-1 Regulation of Chronic Visceral Hyperalgesia" was retracted in 2023. Reasons: signs of a paper mill; compromised peer review; unreliable results or conclusions.

## 3. Results

### 3.1. Characteristics of Experimental Rats

The healthy control group had stronger daily activity, smooth, white hair, formed stool, and normal eating habits. The model group had normal daily activities, slightly rough, and white hair and could eat less than the control group. They occasionally had thin stools, which were easy to provoke. In addition, the model group had stronger responses to the pulling stimulus than the healthy control group. The weights of M group, MC group, F group, and FC group were 153.39 ± 10.18 g, 151.72 ± 9.40 g, 154.86 ± 11.96 g, and 156.63 ± 13.86 g, respectively. There was no difference in weight among groups (Figure 1, *P* > 0.05).

### 3.2. Verification of the Chronic Visceral Hyperalgesia Model

The distension volume threshold causing AWR3 response of the M group, the MC group, the F group, and the FC group before NUCB2/Nesfatin-1 intervention was 4.86 ± 0.12, 3.48 ± 0.18, 4.94 ± 0.17, and 2.80 ± 0.13 mL, respectively. The comparison of the volume of all groups showed no significant difference between the M and F groups, but a significant difference in the other groups (*F* = 707.73, *P* < 0.05). The results showed lower volume threshold in the model group than in the healthy control group (Figure 2), indicating that rats in the model group had higher chronic visceral hyperalgesia sensitivity.

In addition, we observed the pathological changes in the colon tissue of rats in the model group using HE staining. The colon tissue appearance was normal in the model group; there were no obvious dilation, congestion, or other pathological lesions in the intestine. HE staining (Figure 3) showed intact mucosa, submucosa, muscle, and serous layers as well as the villous structure of the colon tissue; a few lymphocytes were occasionally observed. There were no other pathological changes such as inflammation, erosion, ulcers, and abnormal cells.

Finally, we measured the MPO activity of the colon tissue to validate the constructed model. The MPO activity of the colon tissue in the M, MC, F, and FC groups was 0.79 ± 0.18 U/g, 0.81 ± 0.17 U/g, 0.88 ± 1.14 U/g, and 0.82 ± 0.41 U/g, respectively. The comparison of MPO activity among groups showed no significant differences (*F* = 0.0664, *P* > 0.05), indicating the lack of inflammatory reaction of the colon tissue in the model group (Figure 4).

### 3.3. NUCB2/Nesfatin-1 Intervention Led to Different Distension Volume Threshold to Reach AWR Score = 3 among Groups

We evaluated the visceral sensitivity by adopting the minimum distension volume causing AWR3 response as threshold. The results showed lower volume threshold of NUCB2/Nesfatin-1 central intervention groups (MC+NCI group and FC+NCI group; 1.95 ± 0.13 and 1.33 ± 0.05) than NUCB2/Nesfatin-1 peripheral intervention groups (MC+NPI group and FC+NPI group; 2.56 ± 0.17 and 1.66 ± 0.11), confirming that the central intervention group had higher chronic visceral hyperalgesia sensitivity. In the meantime, the liquid volume of the female intervention group was lower than the male intervention group, indicating that the female intervention group had higher visceral sensitivity (Figure 5).

The article "NUCB2/Nesfatin-1 Regulation of Chronic Visceral Hyperalgesia" was retracted in 2023. Reasons: signs of a paper mill; compromised peer review; unreliable results or conclusions.

### 3.4. NUCB2/Nesfatin-1 Intervention Differently Affected the Peak Value of External Oblique Muscle Electrical Activity among Treatment Groups

We evaluated the sensitivity of chronic visceral hyperalgesia using the peak value of the external abdominal oblique muscle electrical activity. The comparison (Figures 6–7) showed that the peak value of NUCB2/Nesfatin-1 central intervention group (MC+NCI group and FC+NCI group; 45.29 ± 1.17 and 50.50 ± 1.52) was higher than that of the NUCB2/Nesfatin-1 peripheral intervention group (MC+NPI group and FC+NPI group; 35.20 ± 2.96 and 40.58 ± 1.74), indicating that the central intervention group had higher chronic visceral hyperalgesia sensitivity. In addition, the peak of the female intervention group was higher than that of the male intervention group, suggesting that the female intervention group had a higher visceral sensitivity.

## 4. Discussion

Chronic visceral hyperalgesia was one of the characteristic mechanisms of discomfort symptoms in IBS, and its occurrence often involved many central and peripheral factors. The effective regulation of chronic visceral hyperalgesia has become the important key which effectively improves the symptoms of IBS [1, 18, 19]. In this study, a chronic visceral hyperalgesia model was built by the central stimulation of maternal separation and the peripheral stimulation of an acetic acid enema. First, we evaluated the general condition of experimental rats. Rats in the model group showed bowel dysfunction symptoms, such as decreased food intake and abnormal defecation. For an equal strength pulling stimulus, female rats in the model group showed a stronger irritability reaction. Second, we adopted the distension volume threshold causing AWR3 response to evaluate visceral sensitivity in model rats [20]. We found that the volume of the model group was lower than that of the healthy control group and that of the FC group lower than the MC group. These results indicated that the model group had higher visceral hyperalgesia sensitivity under stress than healthy controls, a phenomenon consistent with the characteristics of IBS under stress. Finally, the colon tissues of the model group and the healthy control group had normal appearance and color, the colon mucosal structure was intact, and only a few lymphocytes were observed. In the meantime, the MPO activity of colon tissue, which indicates the function and the activity state of neutrophil and could reflect tissue inflammation state, was quantified [21]. The experimental results showed no differences in inflammation between the model and healthy control groups. The present chronic visceral hyperalgesia model simulated the chronic visceral hyperalgesia state of human functional gastrointestinal diseases; it did not affect the growth and weight of experimental rats, and the above parameters indicated successful establishment of the chronic visceral hyperalgesia model.

The article "NUCB2/Nesfatin-1 Regulation of Chronic Visceral Hyperalgesia" was retracted in 2023. Reasons: signs of a paper mill; compromised peer review; unreliable results or conclusions.

NUCB2/Nesfatin-1 plays an important role in multiple signaling pathways in the human body and can regulate digestive tract sensation and movement through various mechanisms [22]. Our previous studies [13] found that NUCB2/Nesfatin-1 could regulate the visceral hyperalgesia sensitivity of male model rats. The results were consistent with the research of Jia et al. [12]. We treated male and female model groups through a central and peripheral approach, respectively. In this study, the distension volume threshold causing AWR3 response and peak value of external oblique muscle electrical activity were chosen to evaluate chronic visceral hyperalgesia sensitivity in behaviorally and electrophysiologically.

From the perspective of behavior, there were no differences in chronic visceral hyperalgesia sensitivity between the MC group, MC+SCI group, MC+SPI group, FC group, FC+SCI group, and FC+SPI group, respectively. This result proved that the central and peripheral approach injection stimulation could not affect chronic visceral hyperalgesia sensitivity. After NUCB2/Nesfatin-1 intervention, the distension volume threshold causing AWR3 response of the MC+NCI group, the MC+NPI group, the FC+NCI group, and the FC+NPI group was lower than in the MC group, the FC group, the MC+SCI group, the MC+SPI group, the FC+SCI group, and the FC+SPI group. These results showed that NUCB2/Nesfatin-1 central and peripheral intervention approaches in both female and male model groups could regulate chronic visceral hyperalgesia sensitivity. In addition, the volume threshold of the MC+NCI group and the FC+NCI group was lower than that of the MC+NPI group and the FC+NCI group, showing that NUCB2/Nesfatin-1 central intervention had a stronger effect than the peripheral intervention. Numerous studies [23–25] have shown that the mechanism of visceral hyperalgesia involves brain center sensitization, facilitation of visceral sensory nerve conduction, sensitization of peripheral receptors, and many other aspects; therefore, the differences caused by NUCB2/Nesfatin-1 central and peripheral intervention on chronic visceral hyperalgesia may be related to a different sensitization degree between NUCB2/Nesfatin-1 upregulated and downregulated signaling pathways, also related to the different sensitization mechanisms. With respect to sex-specific effects, the distension volume threshold causing AWR3 response of the MC group, the MC+NPI group, and the MC+NCI group was lower than that of the FC group, the FC+NPI group, and the FC+NCI group. This result showed higher chronic visceral hyperalgesia sensitivity in the female model group than in the male model group before and after NUCB2/Nesfatin-1 intervention. We speculate that estrogens could increase visceral sensitivity in rats through different intervention approaches (central or peripheral) of NUCB2/Nesfatin-1. Some studies have shown that sex hormones can regulate visceral hyperalgesia and intestinal movement. Estrogen could not only increase of visceral hyperalgesia in female experimental rats, but these changes would periodically follow the physiological cycle of estrogen [26], consistent with the results of our study.

The article "NUCB2/Nesfatin-1 Regulation of Chronic Visceral Hyperalgesia" was retracted in 2023. Reasons: signs of a paper mill; compromised peer review; unreliable results or conclusions.

From the perspective of electrophysiology, the peak value of the MC and FC groups showed no differences compared with the different NUCB2/Nesfatin-1 intervention approaches (MC+SCI group, MC+SPI group, FC+SCI group, and FC+SPI group). This indicated that the peak of external abdominal oblique muscle electrical activity had no effect on the visceral hyperalgesia sensitivity between the different sex MC group and the intervention control group after central and peripheral saline intervention.

Furthermore, we used two different NUCB2/Nesfatin-1 treatment approaches. We found that both central and peripheral treatment with NUCB2/Nesfatin-1 could increase the peak value and cause abnormal external abdominal oblique muscle electrical activity, facilitating the occurrence and conduction of visceral hyperalgesia, ultimately improving visceral hyperalgesia sensitivity. In addition, the peak value in the central intervention group of MC+NCI and FC+NCI groups was higher compared with the peripheral intervention group of MC+NPI and FC+NPI groups; although the chronic visceral hyperalgesia sensitivity also tended to increase, this phenomenon showed that under the same NUCB2/Nesfatin-1 dosage, the central treatment NUCB2/Nesfatin-1 had a stronger effect on the electrical activity of the external oblique muscle than the peripheral intervention. NUCB2/Nesfatin-1 intervention in experimental rats of different sex, the peak value of the MC group, the MC+NPI group, and the MC+NCI group was higher than that of the FC group, the FC+NPI group, and the FC+NCI group. This showed that before or after the same stimulation intervention of NUCB2/Nesfatin-1, Nesfatin-1 increased more chronic visceral hyperalgesia in the female model. However, the specific mechanisms of central and peripheral NUCB2/Nesfatin-1 intervention and how estrogen affects NUCB2/Nesfatin-1 in regulating chronic visceral nociceptive hypersensitivity were not explored in this study. Therefore, it is necessary to further investigate the mechanisms and factors influencing the regulation of chronic visceral nociceptive allergy by NUCB2/Nesfatin-1 at cellular and molecular levels.

The article "NUCB2/Nesfatin-1 Regulation of Chronic Visceral Hyperalgesia" was retracted in 2023. Reasons: signs of a paper mill; compromised peer review; unreliable results or conclusions.

## 5. Conclusion

Our study confirmed that NUCB2/Nesfatin-1 can modulate visceral hyperalgesia in chronic visceral hyperalgesia model rats and that its modulation is related to intervention mode and sex, laying the foundation for exploring strategies to effectively regulate chronic visceral hypersensitivity.

## Figures and Tables

**Figure 1:** Comparison of rat weight among groups. M group: male healthy control group; F group: female healthy control group; MC group: male model control group; FC group: female model control group. *N* = 8 per group.

**Figure 2:** Comparison of distension volume threshold to reach AWR score = 3 among groups before NUCB2/Nesfatin-1 intervention. *N* = 8 per group.

**Figure 3:** Colon tissue HE staining of rats in the model group. Magnification, ×200.

**Figure 4:** Comparison of myeloperoxidase (MPO) activity of colon tissue among groups. *N* = 8 per group.

**Figure 5:** Comparison of distension volume threshold to reach AWR score = 3 among groups after NUCB2/Nesfatin-1 intervention. *N* = 8 per group. ^∗^*P* < 0.05, compared with the MC group; ^#^*P* < 0.05, compared with the FC group. MC group: male model control group; MC+NCI group: NUCB2/Nesfatin-1 central intervention group; MC+SCI group: central intervention control group; MC+NPI group: NUCB2/Nesfatin-1 peripheral intervention group; MC+SPI group: peripheral intervention control group; FC group: female model control group; FC+NCI group: NUCB2/Nesfatin-1 central intervention group; FC+SCI group: central intervention control group; FC+NPI group: NUCB2/Nesfatin-1 peripheral intervention group; FC+SPI group: peripheral intervention control group;

**Figure 6:** Comparison of abdominal withdraw reflex (AWR) = 3 points external oblique muscle electrical activity. *N* = 8 per group. ^∗^*P* < 0.05, compared with the MC group; ^#^*P* < 0.05, compared with the FC group.

The article "NUCB2/Nesfatin-1 Regulation of Chronic Visceral Hyperalgesia" was retracted in 2023. Reasons: signs of a paper mill; compromised peer review; unreliable results or conclusions.

**Figure 7:** External oblique muscle electrical activity in all groups after NUCB2/NUCB2/Nesfatin-1 intervention.

## Data Availability

The data used to support the findings of this study are available from the corresponding author upon request.
